This article has been retracted.

# LncRNA MALAT1 up-regulates VEGF-A and ANGPT2 to promote angiogenesis in brain microvascular endothelial cells against oxygen–glucose deprivation via targetting *miR-145*

**DOI:** 10.1042/BSR20180226

**Published:** 2019-03-06

**Authors:** Lanfen Ren, Chunxia Wei, Kui Li, Zuneng Lu

**Affiliations:** 1 Department of Neurology, Renmin Hospital of Wuhan University, Wuhan 430060, P.R. China; 2 Department of Cardiovascular Surgery, Renmin Hospital of Wuhan University, Wuhan 430060, P.R. China

**Keywords:** BMECs, lncRNA-MALAT1, Stroke

## Abstract

Stroke is one of the leading causes of death and long-term disability around the world. Angiogenesis is supposed to protect brain microvascular endothelial cells (BMECs) from oxidative and ischemic stress. Previous studies indicated that interaction between metastasis-associated lung adenocarcinoma transcript 1 (MALAT1) and *miR-145* was involved in myocardial ischemia reperfusion, suggesting MALAT1 and *miR-145* were also mediated with the progress of angiogenesis and cell migration in oxygen–glucose deprivation (OGD)-induced BMECs. The present study aimed to investigate the functional roles of MALAT1 in regulating *miR-145* and its downstream pro-angiogenesis factors, vascular endothelial growth factor (VEGF)-A and Angiopoietin-2 (ANGPT2) during the progress of angiogenesis in OGD-induced BMECs. An *in vitro* OGD model was employed in mouse BMECs to mimic brain hypoxic and ischemic conditions; MTT was used to determine cell viability. qRT-PCR was used to determine the expression of long non-coding RNA (lncRNA)-MALAT1 and *miR-145* under OGD conditions; *in vitro* tube formation assay was used to investigate angiogenic effect of MALAT1 and *miR-145*. The relationship between lncRNA-MALAT1/*miR-145* and *miR-145*/VEGF-A/ANGPT2 was evaluated by qRT-PCR and Western blot, and direct binding was assessed using dual luciferase assay. Results showed that the levels of lncRNA-MALAT1 and *miR-145* were up-regulated in OGD-induced BMECs. *miR-145* functioned as an anti-angiogenic and pro-apoptotic factor in OGD treated BMECs via down-regulating VEGF-A and ANGPT2 directly. While lncRNA-MALAT1 enhanced the expressions of VEGF-A and ANGPT2 by targetting *miR-145* to promote angiogenesis and proliferation of BMECs under OGD conditions. Our present study revealed the inhibitory functions of *miR-145* on angiogenesis through direct targetting on VEGF-A and ANGPT2 for the first time and proved the protective role of lncRNA-MALAT1 for BMECs under OGD conditions through the direct regulation of *miR-145*.

## Introduction

Stroke is reported to be one of the major diseases leading to deaths worldwide, which is accompanied with symptoms such as cerebral ischemia or hypoxia. Ischemic stroke which accounts for over 80% of all the stroke cases in addition to hemorrhagic stroke, is the consequence of thrombotic or embolic occlusion of major cerebral arteries [1], which is the predominant cause of long-term disability [2]. Current strategies to treat patients suffering from ischemic stroke include recanalization and neuroprotective strategies. The administration of intravenous recombinant tissue-type plasminogen activator (tPA) to establish revascularization, use of intra-arterial fibrinolysis, or mechanical clot retrieval is common in recanalization strategies, while the effectiveness of this type of treatment highly relies on the time period in which it is administrated [3]. Neuroprotective strategies are implemented to preserve the penumbral tissues as well as extending the time window for revascularization treatment. However, neuroprotection was shown to insufficient to treat stroke due to the lack of clinical effectiveness [4]. Possible reasons may include the complexity of interplays in multiple pathways, the acute cerebral injury/neurological impairments following ischemia, and the lack of defining treatments for specific targets [5].

Angiogenesis is an important process in which new microvessels sprouting from the existing vascular endothelial cells that release from extracellular matrix and migrate to further differentiate into new blood tubule [6]. The process of angiogenesis is regulated by the interplay of multiple pro-angiogenic and anti-angiogenic factors [7]. It is considered that angiogenic sprouting can provide essential oxygen and nutrition supply for the development of disseminated cells [8]. Evidence indicates that the barrier function of brain microvascular endothelial cells (BMECs), the first type of neurovascular to sense hypoxia stimulation, can be disrupted after cerebral ischemic injury and cause a vascular leakage [9]. Function recovery was observed when angiogenesis was promoted after hypoxia/ischemia injury, and was correlated to a better prognosis of patients who suffered from cerebral ischemia clinically [10–12]. Hence, the induction of angiogenesis in BMECs under hypoxic stress could be a potential neuroprotective way to treat ischemic stroke.

Non-coding RNAs have been elucidated to be functionally involved in mechanisms of angiogenesis, carcinogenesis, and metastasis [7]. Long non-coding RNAs (lncRNAs) refer to those which are more than 200 nts in length. The repressive function of lncRNA on the expression of miRNA through the competing mechanism potentially explains the significance of studying the interplays of lncRNA and miRNA in related fields [13]. Based on the recent study of altered lncRNA transcriptomic profiles in brain microvascular endothelium after cerebral ischemia [14], the metastasis-associated lung adenocarcinoma transcript 1 (MALAT1) was verified as one of the most up-regulated lncRNAs, which was involved in protecting BMECs from cerebral ischemic injury [15]. Additionally, the underlying mechanism of the protective role of MALAT1 in BMECs against ischemic cerebral injury is thought to be mediated by the induction of moderate autophagy, which makes it an interesting target [16]. Notably, MALAT1 was demonstrated to act as an anti-apoptotic and anti-inflammatory factor in cerebral microvasculature after ischemic cerebral vascular and parenchymal damages [16]. However, whether MALAT1 prevents oxygen–glucose deprivation (OGD)-induced brain cell damage through promoting angiogenesis still remains unclear.

Mounting studies suggest that *miR-145* is up-regulated by hypoxia and facilitates hypoxia-induced cell injury [18]. Earlier findings on the suppressive role of *miR-145* in angiogenesis through mediating the expressions of vascular endothelial growth factor (VEGF) and Angiopoietin-2 (ANGPT2) in cancers suggests that a possible regulatory pathway may exist in the physiological progress of ischemic stroke as well [19,20]. VEGF-A, which belongs to VEGF family, is a permeability factor in angiogenesis progress [21]. It has attracted growing attention due to cross-talk between its regulatory role in new blood vessel formation and neurones. Both pro-VEGF and anti-VEGF therapies have been implemented in ischemic stroke, and the rescue and edematous effects caused by VEGF therapy have been reported during the clinical treatment. However, the effects of usage of VEGF are highly dependent on the concentration, timing, and source of VEGF [22]. ANGPT2 is a member of angiopoietin family and exists mostly in cells requiring vascular remodeling. As ANGPT2 is crucial in switching on tyrosine kinase receptors TIE2 (EC membrane receptor) pathway, it is highly associated with predisposition of cellular angiogenesis status, and is a current target for anti-angiogenic drugs [23].

Given that *miR-145* and MALAT1 directly bind and reciprocally inhibit each other [24], here, we proposed the hypothesis that MALAT1 up-regulates VEGF-A and ANGPT2 through inhibiting *miR-145*, and eventually facilitates angiogenesis in mouse BMECs under hypoxic/ischemic conditions.

## Materials and methods

### Isolation of BMECs and primary culture

Twenty male C57BL/6J mice (25–30 g in body weight, 3–4 months old) were purchased from the Shanghai Laboratory Animal Center (Shanghai, P.R. China) and were fed *ad libitum* before experiments. According to previously reported methods, mice were anesthetized with an intraperitoneal injection of 40 mg/kg pentobarbital and then killed by cervical dislocation before isolation of cerebral cortex. The extracted cerebral cortex was treated in ice-cold HBSS added with antibiotics to discard meninges and superficial blood vessels. Gray matters were obtained after homogenizing and filtering the cerebral cortex, followed by digestion with 4 mg/ml collagenase B and 1 mg/ml collagenase/dispase (Roche Molecular Biochemicals, Indianapolis, IN) for 2 h sequentially and then centrifuged in 40% Percoll solution [25]. The second band containing microvessels was collected and washed to plate on to collagen-coated dishes. Cells that migrated from the microvessels were collected to be cultured in DMEM containing 10% FBS, 75 μg/ml endothelial cell growth supplement, and 0.5 mg/ml heparin. Mouse BMECs of 1–5 passages that were positive for factor VIII and Vimentin indicated >95% endothelial cell purity and were selected by bradykinin receptors. Then BMECs were cultured to 85–95% confluence before use. All procedures and animal care were approved by the Committee of Animal Care in accordance with National Institutes of Health Guidelines. Five mice were used in each isolation and culture, and the primary culture was repeated for three times.

### Application of OGD model

In order to mimic hypoxic/ischemic conditions *in vitro*, an OGD model was deployed here based on previously mentioned method [26]. BMECs were cultured in 95% N_2_/5% CO_2_ (deoxygenated) and glucose-free conditions in hypoxic chambers for indicated time.

### Cell transfection

siRNA was used to knockdown the expression of MALAT1; pcDNA-MALAT1 was used to amplify the expression of MALAT1. The full-length cDNA of human MALAT1 was amplified using the following primer sets: 5′-GGCGGTACCATGAAACAATTTGGAGAAG-3′ (forward) and 5′-GCGCTCGAGCTAAGTTTGTACATTTTGCC-3′ (reverse). The cDNA was subsequently cloned into pcDNA mammalian expression vector (Invitrogen) in order to generate pcDNA-MALAT1 stable colonies. The pcDNA vector was used as negative control (pcDNA-control). For MALAT1 knockdown, a MALAT1-targetting siRNAs kit (GenePharm, Shanghai, P.R. China) was used to silence the expression of MALAT1 (si-MALAT1). A scrambled negative control (GenePharm, Shanghai, P.R. China) was used as negative control (si-control). *miR-145* mimic and inhibitor were deployed to change the expression level of *miR-145* in BMECs. Two control miRNAs (*mimic-NC* and *inhibitor-NC*) (GenePharm, Shanghai, P.R. China) were used as negative controls for *miR-145* mimic and *miR-145* inhibitor, respectively. The constructed si-MALAT1, pcDNA-MALAT1, *miR-145* mimic/*miR-145* inhibitors were transfected into BMECs using Lipofectamine 2000 (Invitrogen, CA, U.S.A.) according to the manufacturer’s instructions.

### MTT assay

MTT assay was used to evaluate the survival of BMECs with OGD treatment. BMECs were plated at 10000 cells per cm^2^ in 96-well plates, added with 20-µl MTT (Sigma–Aldrich, St. Louis, U.S.A.) per well. The plate was then incubated for 4 h at 37°C. The supernatant was collected and the cell layer was dissolved in 150-µl DMSO. To solubilize crystals, the plate was shaken for 15 min and the optical density of each well was determined using a model 680 microplate reader at 490 nm (Bio-Rad, Hercules, U.S.A.).

### Transwell assay

Cell migration was assayed using a Transwell chamber (Millipore, MA, U.S.A.). BMECs (5  ×  10^4^) in 250-μl DMEM were added into the upper chamber. And 500-μl DMEM containing 10% FBS was added to the lower chamber. BMECs underwent starvation before incubation at 37°C for 24 h. Then the cells on the upper side of well were scraped off. The migrated cells were fixed with methanol for 20 min and followed by staining using Crystal Violet for 20 min. Images were obtained under a phase-contrast microscope (Olympus, Japan).

### Tube formation

Matrigel plug assay was used to measure angiogenesis based on protocol mentioned previously [27]. Briefly, 2 × 10^6^ cells in 400 μl solution containing 80% Matrigel were injected subcutaneously. Plug was then harvested for 4 days, weighed, and photographed. Plug was dispersed in 400 μl of PBS in order to collect the hemoglobin. Hemoglobin content was measured using Drabkin’s solution (Sigma, Missouri, U.S.A.) according to manufacturer’s recommendations.

### Western blot analysis

BMECs were harvested 48 h after transfection and lyzed in Triton X-100 lysis buffer for 30 min at 4°C; 50 μl of whole cell lysates were separated using SDS/PAGE and electrophoretically transferred on to PVDF membranes. The membrane was incubated with primary antibody against VEGF-A (Cell Signaling Technology, MA, U.S.A.) and ANGPT2 (Cell Signaling Technology, MA, U.S.A.) for 20 h at 4°C. The membrane was then washed and stained with respective horseradish peroxidase conjugated secondary antibodies (Alexa Fluor; Molecular Probes, Eugene, U.S.A.) for 1 h at room temperature. Protein bands were visualized using ECL and signals were detected using the ECL detection system (Thermo Fisher Scientific).

### Quantitative real-time PCR

Total RNA samples from BMECs were extracted using TRIzol reagent (Invitrogen, Carlsbad, U.S.A.) according to the manufacturer’s instructions. The concentration of isolated total RNA was measured using NanoDrop ND-1000 spectrophotometer (Agilent, CA, U.S.A.). Then 0.5 μg of RNA was reverse-transcribed using high-capacity cDNA reverse transcription kit (Applied Biosystems, Foster City, U.S.A.) to obtain first-strand cDNA. Specifically, *miR-145* expression level was quantitated using mirVana qRT-PCR miRNA detection kit (Ambion, Austin, U.S.A.) in conjunction with SYBR Green PCR Kit (Thermo Fisher Scientific, MA, U.S.A.) with 7500 real-Time PCR system (Applied Biosystems, CA, U.S.A.). The target gene expression was normalized to snRNA U6. Primers used for *miR-145*: 5′-GCCGCGTCCAGTTTTCCCAGG-3′ (forward) and 5′-GTGCAGGGTCCGAGGT-3′ (reverse); MALAT1: 5′-AGACCTTGAAATCCAT-3′ (forward) and 5′-CTTCTGCTTCCTACTT-3′ (reverse); U6: 5′-CTCGCTTCGGCAGCACA-3′ (forward), 5′-AACGCTTCACGAATTTGCGT-3′ (reverse). VEGF-A: 5′-GCTGTCTTGGGTGCATTGGA-3′ (forward) and 5′-ATGATTCTGCCCTCCTCCTTCT-3′ (reverse); ANGPT2: 5′-CCGCTACGTGCTTAAGATCC-3′ (forward) and 5′-ATTGTCCGAATCCTTTGTGC-3′ (reverse).

### Dual-luciferase reporter assay

The 3′-UTR of *MALAT1, VEGF-A*, and *ANGPT2* genes containing the predicated binding sites for *miR-145* were amplified using PCR. The fragment was inserted into the multiple cloning sites in the pMIR-REPORT luciferase miRNA expression reporter vector (Ambion, Austin, U.S.A.). Then BMECs were co-transfected with 0.1 µg of luciferase reporter vectors comprising wild-type or mutant-type of 3′-UTR of MALAT1, VEGF-A, or ANGPT2 and either *miR-145* mimic or miR-control by Lipofectamine 2000 (Invitrogen, Carlsbad, U.S.A.). Relative luciferase activity was calculated by normalizing the firefly luminescence to the *Renilla* luminescence using the Dual-Luciferase Reporter Assay System (Promega, Madison, WI, U.S.A.) according to the manufacturer’s instructions at 48 h post-transfection.

### Statistical analysis

Data were presented as the means ± S.D. based on at least three independent experiments. Data amongst multiple groups were analyzed using one-way ANOVA and followed by Tukey *post hoc* tests for multiple comparisons. The standard two-tail Student’s *t* test was used to determine statistical significance for comparison between two groups. *P*<0.05 was considered statistically significant. Statistical analysis was performed using SPSS 17.0 software (SPSS, Chicago, IL, U.S.A.).

## Results

### OGD attenuated the viability of BMECs and elevated expression of lncRNA-MALAT1 and *miR-145*

The effect of OGD treatment on cell viability of mice BMECs were evaluated over a timecourse of 24 h by MTT assay. Figure 1A illustrates that the viability of mice BMECs was significantly attenuated following the longer OGD treating time, suggesting injury of BMECs was caused under hypoxic/ischemic conditions. qRT-PCR results indicated that expression of MALAT1 and *miR-145* increased to approximately six-fold and five-fold compared to that under normoxic conditions, respectively during 24 h OGD treatment (Figure 1B,C).

**Figure 1:** OGD treatment attenuated cell viability of BMECs and up-regulated expression of lncRNA-MALAT1 and *miR-145* (**A**) MTT assay measured the viability of mouse BMECs after OGD treatment for 0, 6, 12, and 24 h. (**B**) qRT-PCR analysis of lncRNA-MALAT1 expression level in OGD (0, 6, 12, 24 h) treated BMECs. (**C**) qRT-PCR analysis of *miR-145* expression level in OGD (0, 6, 12, 24 h) treated BMECs. Data represent means ± S.D. based on three independent experiments; *P<0.01, **P<0.05.

### LncRNA-MALAT1 promoted angiogenesis and migration in BMECs under OGD stimulation

LncRNA-MALAT1 was confirmed to be stably knocked down or overexpressed in BMECs (Figure 2A). The effects of lncRNA-MALAT1 on BMECs tubule formation under OGD conditions (12 h) were assessed as Figure 2D shows microtubule formation was overall weakened in mice BMECs cultured under OGD conditions for 12 h. Specifically, total tubule density was increased when MALAT1 was overexpressed, and decreased when MALAT1 was silenced. Quantitative analysis illustrated that tube length decreased by approximately 50% under the OGD conditions compared with that under normoxic conditions. New sprout tubes were truncated approximately 25% in si-MALAT1 group compared with that in si-control, while a 50% increase in tube length was observed in MALAT1 overexpression group compared with that in pcDNA-control (*P*<0.05) (Figure 2B). As shown in Figure 2C,E, the number of migrated BMECs under OGD conditions decreased 55% compared with that under normoxic conditions. Likewise, a reduction of 55% in migrated BMECs was observed in si-MALAT1 group compared to that in si-control, while the quantity of migrated cells increased to approximately 2.1-fold when MALAT1 was overexpressed (*P*<0.05). Moreover, we found that MALAT1 knockdown significantly elevated mir-14 expression (Figure 3C).

**Figure 2:** LncRNA-MALAT1 promoted angiogenesis of mouse BMECs under OGD conditions (**A**) qRT-PCR test of stable lncRNA-MALAT1 overexpression in pcDNA-MALAT1 group and lncRNA-MALAT1 knockdown in si-MALAT1 group. (**B**) The results of tubule formation in groups mentioned in (A) were expressed as relative tube length. (**C**) Migration of BMECs was measured by Transwell migration assay and presented in the form of number of migration cells. (**D**) The effects of lncRNA-MALAT1 on tube formation in BMECs was measured by Matrigel assay. (**E**) The results of migrated BMECs under OGD stimulation were expressed as the number of migrated cells per field (magnification: ×200; scale bar: 100 μm). BMECs were treated under OGD conditions for 12 h, grouping as OGD(−), OGD(12 h), si-control, si-MALAT1, pcDNA-control, and pcDNA-MALAT1. Data represent means ± S.D. based on three independent experiments; *P<0.05, **P<0.01.

### LncRNA-MALAT1 up-regulated VEGF-A and ANGPT2 via targetting *miR-145*

The effects of lnc-MALAT1 on the expression of pro-angiogenesis factors VEGF-A and ANGPT2 were evaluated using qRT-PCR and Western blot. As shown in Figure 3A,B, a trend of relative expression level was consistent in terms of VEGF-A and ANGPT2 to increase under OGD conditions compared with that under normoxic conditions. Pro-angiogenesis factors mentioned above were down-regulated in si-MALAT1 group (for VEGF-A approximately 50%, for ANGPT2 approximately 37.5%) compared to that in si-control group, while up-regulated in pcDNA-MALAT1 group (for VEGFA approximately two-fold, for ANGPT2 approximately 2.1-fold) compared to that in pcDNA-control group. Results of the Western blot were consistent with that of qRT-PCR (Figure 3D).

**Figure 3:** LncRNA-MALAT1 up-regulated VEGF-A and ANGPT2 via targetting *miR-145* (**A**) qRT-PCR analysis was performed to measure relative expression level of VEGF-A in BMECs. (**B**) qRT-PCR analysis was performed to measure relative expression level of ANGPT2 in BMECs. (**C**) qRT-PCR analysis was used to measure the effects of MALAT1 on the expression level of *miR-145* in BMECs. (**D**) Western blot analysis was performed to measure protein levels of VEGF-A and ANGPT2, GAPDH was used as an internal control. (**E**) Conservation of MALAT1 at the binding site of *miR-145* was snapshot, 5 nts on 3′-UTR of MALAT1 were replaced in constructed MALAT1 mutant. (**F**) Dual-luciferase reporter assay was used to measure relative luciferase activity. BMECs were treated under OGD conditions for 12 h, grouping as OGD(−), OGD(12 h), si-control, si-MALAT1, pcDNA-control, and pcDNA-MALAT1. Data represent means ± S.D. based on three independent experiments; *P<0.05, **P<0.01.

The dual luciferase reporter system was constructed to validate the interplay of MALAT1 and *miR-145*. The potential binding sequence of *miR-145* was predicted by the bioinformatics database (Figure 3E). As Figure 3F shows, the relative luciferase activity decreased by over 70% in cells co-transfected with MALAT1 wild-type and *miR-145* mimic (*P*<0.01), while no significant difference was observed in cells co-transfected with MALAT1 mutant and *miR-145* mimic, compared with mimic NC. Furthermore, the level of *miR-145* in BMECs was validated to be up-regulated after OGD treatment (12 h) compared with that under normoxic conditions (*P*<0.05). The expression of *miR-145* increased two-fold in si-MALAT1 group compared to that in si-control group (*P*<0.01), but decreased two-fold in pcDNA-MALAT1 group compared to that in pcDNA-control group (*P*<0.05).

### *miR-145* suppressed angiogenesis and migration in BMECs under OGD stimulation

The efficacy of *miR-145* knockdown and overexpression was validated (Figure 4A) using qRT-PCR. The relative tube length decreased by 50% under the OGD conditions compared with that under normoxic conditions (*P*<0.05). New sprout tubes were truncated by 50% in *miR-145* mimic group compared with that in mimic NC group (*P*<0.05); conversely a two-fold increase in tube length was observed in *miR-145* inhibitor group compared with that in inhibitor NC group (*P*<0.05) (Figure 4B,D). According to the results of the Transwell assay shown in Figure 4C,E, the migration of BMECs was significantly suppressed in OGD group (12 h) compared to that in normoxic group. Migrated cells increased two-fold in the *miR-145* inhibitor group compared to that in inhibitor control group (*P*<0.05), while the number decreased two-fold in *miR-145* mimic group compared to that in mimic control group (*P*<0.05).

**Figure 4:** *miR-145* inhibited angiogenesis and cell migration in BMECs under OGD conditions (**A**) qRT-PCR analysis was used to verify the stability of *miR-145* knockdown or overexpression. (**B**) The results of Matrigel assay were plotted as relative tube length. (**C**) The results of migrated BMECs under OGD stimulation were expressed as the number of migrated cells per field (magnification: ×200; scale bar: 100 μm). (**D**) Matrigel assay was used to evaluate the effects of *miR-145* on angiogenesis in BMECs. (**E**) Migration of BMECs was measured by Transwell migration assay. BMECs were treated under OGD conditions for 12 h, grouping as OGD(−), OGD(12 h), mimic NC, *miR-145* mimic, inhibitor NC, and *miR-145* inhibitor. Data represent means ± S.D. based on three independent experiments; *P<0.05, **P<0.01.

### *miR-145* suppressed expression of VEGF-A and ANGPT2 via targetting 3′-UTR sites

The effects of *miR-145* on the expression levels of pro-angiogenesis factors VEGF-A and ANGPT2 were evaluated using qRT-PCR and Western blot, and the reciprocal interactions were analyzed using dual-luciferase reporter assay. Expressions of VEGF-A and ANGPT2 decreased approximately 50% in *miR-145* mimic group compared to that in mimic control group (*P*<0.05), while increased approximately two-fold in *miR-145* inhibitor group compared to that in inhibitor control group (Figure 5A,B) (for VEGF-A *P*<0.01, for ANGPT2 *P*<0.05). The overall expressions of VEGF-A and ANGPT2 were elevated after OGD treatment (12 h) compared to that under normoxic conditions. Western blot assay revealed similar trends amongst groups (Figure 5C).

**Figure 5:** *miR-145* attenuated VEGF-A and ANGPT2 in BMECs under OGD conditions (**A**) qRT-PCR analysis was performed to measure relative expression level of VEGF-A in BMECs. (**B**) qRT-PCR analysis was performed to measure relative expression level of ANGPT2 in BMECs. (**C**) Western blot analysis was performed to measure protein levels of VEGF-A and ANGPT2. GAPDH was used as an internal control. BMECs were treated under OGD conditions for 12 h, grouping as OGD(−), OGD(12 h), mimic NC, *miR-145* mimic, inhibitor NC, and *miR-145* inhibitor. Data represent means ± S.D. based on three independent experiments; *P<0.05, **P<0.01.

The interplay between *miR-145* and VEGF-A/ANGPT2 was assessed using dual-luciferase reporter system subsequently. Figure 6 illustrates the nucleotides in 3′-UTR of *VEGF-A/ANGPT2* mRNA containing a putative binding site, which is a complementary sequence of the seed region of *miR-145* (Figure 6A). The relative luciferase activity decreased over 70% in cells co-transfected with VEGF-A wild-type and *miR-145* (*P*<0.01), yet no significant difference was observed in VEGF-A mutant and *miR-145* group (Figure 6B). Cell lines co-transfected with wild-type 3′-UTR of ANGPT2 and *miR-145* demonstrated over 70% lower luciferase activity compared with mimic NC group while no significant difference was observed in the two groups transfected with mutant 3′-UTR of ANGPT2 (Figure 6C) (*P*<0.01).

**Figure 6:** *miR-145* targetted 3′-UTR of VEGF-A and ANGPT2 (**A**) The luciferase reporter constructs containing the wild-type (WT) or mutant (MUT) 3′-UTR of ANGPT2 or VEGF-A. (**B**) Wild-type VEGF-A or mutant VEGF-A was co-transfected into 293T cells with *miR-145* or mimic NC. (**C**) Wild-type ANGPT2 or mutant ANGPT2 was co-transfected into 293T cells with *miR-145* or mimic NC. Luciferase activity was determined at 48 h after transfection. Data represent means ± S.D. based on three independent experiments; **P<0.01.

## Discussion

In the present study, the expressions of both lncRNA-MALAT1 and *miR-145* were confirmed to be up-regulated under hypoxic conditions. The results demonstrated that lncRNA-MALAT1 promoted angiogenesis in mouse BMECs and played an important role in microtubule formation as well as BMEC migration via up-regulating the expressions of pro-angiogenic factors VEGF-A and ANGPT2. *miR-145* was shown to suppress angiogenesis in BMECs and down-regulate the expressions of pro-angiogenesis factors mentioned above through targetting their 3′-UTR regions. Additionally, MALAT1 was validated to inhibit *miR-145* via direct binding.

Previous studies have demonstrated the roles of angiogenesis in tumor cell formation and metastasis, for it promotes cell survival against environmental stresses such as hypoxia, ischemia, or the reduction in nutrients through up-regulating several pro-angiogenesis factors including VEGF and ANGPT2 [28,29]. Given that function recovery was observed in BMECs that underwent ischemic injury where angiogenesis was promoted [10,12], the induction of angiogenesis in brain tissues injured by hypoxic/ischemic damages may provide new insights into treating ischemic stroke. Recent studies have defined the simulative functions of lncRNA-MALAT1 in the biological process of angiogenesis in several cancers [30–32] as well as its role in the induction of moderate BMEC autophagy against hypoxia/ischemic conditions [33]. In the present study, we investigated the potential role of lncRNA-MALAT1 in regulating angiogenesis progress of BMECs under OGD conditions. Our findings are in accordance with the previous study that lncRNA-MALAT1 was significantly up-regulated in mouse BMECs under OGD conditions [16]. Of note, we confirmed lncRNA-MALAT1 can promote angiogenesis progress in OGD-induced BMECs based on the results of *in vitro* microtubule formation assay and the subsequent cell migration assay. It also suggested that the facilitative function of IncRNA-MALAT1 is dependent on up-regulating VEGF-A and ANGPT2.

To further uncover the underlying molecular mechanism of how lncRNA-MALAT1 regulated the expressions of VEGF-A and ANGPT2, the role of *miR-145* was investigated in the present study. *miR-145* was also confirmed to be up-regulated in BMECs that underwent OGD treatment, which is in-line with the recent finding [18]. This is the first time that *miR-145* has been demonstrated to inhibit angiogenesis progress in BMECs treated by OGD in addition to showing its potential to attenuate cell proliferation. This finding is supported by a recent study that suggests that *miR-145* aggravates hypoxia-induced damage [18]. Moreover, it is consistent with previous findings that *miR-145* was demonstrated to inhibit angiogenesis through regulating pro-angiogenesis factors VEGF-A and ANGPT2 [19,20]. miRNA was previously reported to competitively bind to lncRNA and to get involved in pro-/anti-angiogenesis in several biological processes, specifically, *miR-145* cluster was proved to act as an angiogenesis blocker [34]. An earlier study elucidated the reciprocally inhibitory regulation between *miR-145* and lncRNA-MALAT1 in human endothelial progenitor cells [24]. Here, our findings confirmed that lncRNA-MALAT1 can down-regulate the expression of *miR-145* via direct targetting. Collectively, *miR-145* is suggested to inhibit angiogenesis through directly down-regulating VEGF-A and ANGPT2, and lncRNA-MALAT1 regulated the expression of VEGF-A and ANGPT2 via targetting *miR-145* in OGD-induced mouse BMECs.

However, limitations still exist in the current study. As *in vitro* experiments were implemented in the mouse BMECs, the real cerebral microenvironments could not be fully mimicked. Hence the potential influences of inflammation and edema on lncRNA-MALAT1/VEGF-A/ANGPT2/*miR-145* regulatory axis was not included in the present study. Although angiogenic factors were revealed as a pathological contributor in tumorigenesis due to their roles in facilitating angiogenesis and promoting metastasis, other recent studies indicated double side effects of pro-angiogenesis factors in the physiological path of stroke especially for VEGF [22]. VEGF was reported to induce endothelial permeability which can damage BBB [35], and this function is highly age- and dose-dependent, and the dynamic regulation between VEGF and its receptor VEGFR2 is a considerable factor to be highlighted in complicated pathophysiology [36]. Further investigation should be done to confirm whether the function of MALAT1 has a double edge or if there is another downstream protective signal regulated by MALAT1. In addition, further studies are required as only young adult mice BMECs were involved in the present study, which may cause discrepancy compared with the clinical reality as the age-related altered levels of angiogenic factors could impact the complex brain microenvironments in human. The experiments on related epigenetic and genetic interactions are hence needed to be performed in human brain endothelial microvascular cells to further validate its functions in patients suffering from stroke. Additionally, potential influences of other signaling pathways such as EGFR/Erb [37] on regulating neurovascular networks should be considered in future studies.

In summary, our study suggests that lncRNA-MALAT1 may function as a protective factor in stroke pathophysiology by induction of angiogenesis in brain vascular endothelium, thus maintaining the integrity of brain–blood barrier, which is meaningful in stability of neurone network. The present study defines for the first time the regulatory functions of lncRNA-MALAT1 and *miR-145* on the expression of VEGF-A and ANGPT2 in addition to their direct effects on regulating angiogenesis progress in BMECs under OGD conditions. Our study indicates that the up-regulation of lncRNA-MALAT1 may function to down-regulate *miR-145*, which further induces VEGF-A/ANGPT2 levels in OGD-induced BMEC. These findings provide us with a better understanding on the pathophysiology of stroke and contribute to studies on the novel therapeutic targets of stroke.

## Abbreviations

ANGPT2: angiopoietin-2
BMEC: brain microvascular endothelial cell
lncRNA: long non-coding RNA
MALAT1: metastasis-associated lung adenocarcinoma transcript 1
OGD: oxygen–glucose deprivation
VEGF: vascular endothelial growth factor
